RETRACTED

# Magnetic resonance imaging and ^18^F-fludeoxyglucose positron emission tomography/computed tomography findings of retroperitoneal clear cell carcinoma with an unknown primary site: A case report

**DOI:** 10.3389/fmed.2022.1024008

**Published:** 2022-11-01

**Authors:** Dao-Bing Zeng, Chan Chang, Xu-Sheng Liu, Yan Gao, Ya-Lan Wang, Zhi-Jun Pei

**Affiliations:** ^1^Department of Nuclear Medicine, Taihe Hospital, Hubei University of Medicine, Shiyan, China; ^2^Department of Respiratory and Critical Care Medicine, Taihe Hospital, Hubei University of Medicine, Shiyan, China

**Keywords:** ^18^F-FDG PET/CT, MRI, clear cell carcinoma, retroperitoneum, kidney, pathology

## Abstract

Herein, we report a case of retroperitoneal clear cell carcinoma (RCCC) with an unknown primary site that was confirmed *via* pathology. A 46-year-old man presented with low-grade fever, hyperhidrosis, and nightly fatigue that had occurred for the last 20 days. His weight had decreased significantly within the past 2 months (approximately 12 kg). On abdominal ultrasound, a mass was observed near the left renal hilum. In addition, enhanced magnetic resonance imaging (MRI) of the abdomen revealed a retroperitoneal nodular mass; however, no abnormalities in either kidney or adrenal glands were observed. ^18^F-fludeoxyglucose positron emission tomography/computed tomography (^18^F-FDG PET/CT) demonstrated an intensely FDG-avid retroperitoneal mass, the maximum standardized uptake value (SUVmax) was 19.6. On March 8, 2021, left retroperitoneal lesion resection, retroperitoneal lymph node dissection, and double kidney exploration were performed under general anesthesia. A post-operative pathological examination revealed Poorly differentiated clear cell carcinoma (left retroperitoneal) and metastatic lymph nodes. Immunohistochemical findings showed that the tumor originated from the kidney. At 6-month follow-up, reexamination of the patient revealed retroperitoneal lesion recurrence; however, no abnormalities were observable *via* enhanced computed tomography (CT) of both kidneys. To our knowledge, there have been no previous reports of RCCC of unknown origin.

## Introduction

Approximately 80% of all primary renal cell carcinomas are clear cell carcinomas, making them the most common pathological type of renal cell carcinoma (1). Nonetheless, reports of retroperitoneal clear cell carcinoma (RCCC) are extremely rare. There have been no previous reports on this subject in the literature. Herein, we report a case of RCCC that was pathologically confirmed. Although immunohistochemistry suggested the carcinoma was renal in origin, no obvious abnormality was found *via* imaging or the surgical exploration of both kidneys.

RETRACTED

## Manuscript formatting

### Headings

#### Case presentation

A 46-year-old male who had experienced fever of unknown cause for the past 20 days presented with fever at night, night sweats, and a slight sense of fatigue. After sweating, the patient’s body temperature returned to normal in the morning. A routine blood examination at an external hospital revealed elevated C-reactive protein and ESR levels of 28.0 mg/L (normal value 0–10 mg/L) and 25.0 mm/h (normal value 0–15 mm/h), respectively. Abdominal color ultrasound and enhanced computed tomography (CT) findings suggested retroperitoneal space-occupying lesions. The patient had no known history of malignancy. After admission, a magnetic resonance imaging (MRI) of the upper abdomen was performed. MRI findings indicative of the retroperitoneal mass were as follows (Figure 1). In addition, MRI suggested that retroperitoneal mass may be a metastatic tumor.

**FIGURE 1:** Magnetic resonance imaging (MRI) findings. Low signal on T1WI and heterogeneously high signal on T2WI [**(A,B)**, arrows], and high signal on axial diffusion-weighted imaging [DWI, B600; **(C)**, arrow] indicate the presence of a retroperitoneal mass. Axial early arterial and portal venous post-contrast T1-weighted fat-suppressed imaging findings indicating a heterogeneously enhanced mass are shown [**(D,E)**, arrows]; Retroperitoneal mass enhancement is more obvious in the delayed post-contrast T1-weighted fat-suppressed image [**(F)**, arrow].

A whole body ^18^F-fludeoxyglucose positron emission tomography/computed tomography (^18^F-FDG PET/CT) (Figure 2) was performed to identify primary malignancy, PET/CT images demonstrated a retroperitoneal soft tissue density mass with Significantly increased FDG activity (SUVmax: 19.6), and revealed a lymph node adjacent to the mass with elevated FDG uptake (SUVmax: 7.9).^18^F-FDG PET/CT did not detect potential tumors in other parts of the body. After imaging, the patient underwent a percutaneous biopsy guided by color ultrasound. A percutaneous retroperitoneal mass biopsy revealed a poorly differentiated carcinoma with immunohistochemical findings indicating it may have been renal in origin. Four weeks later, left retroperitoneal lesion resection, retroperitoneal lymph node dissection, and double kidney exploration were performed under general anesthesia. A post-operative pathological examination (Figure 3A) indicated clear cell carcinoma (left retroperitoneal) and metastatic lymph nodes. The following immunohistochemical findings (Figure 3B) suggested the carcinoma was renal in origin: Ki-67 (approximately 30% +), PAX8 (+), CK8 (+), vimentin (+), and PLAP (weak +). No abnormalities were found on imaging and intraoperative exploration of both kidneys in this case. On 6-month follow-up, abdominal enhanced CT revealed retroperitoneal lesion recurrence (Figure 4); however, there remained no obvious abnormality in either kidney.

RETRACTED

**FIGURE 2:** Whole body ^18^F-fludeoxyglucose positron emission tomography/computed tomography (^18^F-FDG PET/CT) as a screen for primary malignancy. An axial computed tomography (CT) image demonstrating a retroperitoneal soft tissue density mass at the level of the left hilum is shown in **(A)** (arrow). PET **(B)**, fused PET/CT images **(C)**, and a maximum intensity projection (MIP) image **(G)** revealing significantly increased FDG activity in the left retroperitoneal mass (arrow) are shown. An axial CT image **(D)** reveals the presence of a lymph node adjacent to the mass (arrow), while PET **(E)** and fused **(F)** images show significant uptake of FDG by the retroperitoneal lymph node.

**FIGURE 3:** Pathological and immunohistochemical (IHC) findings. Post-operative pathological findings **(A)** reveal clear cell carcinoma (left retroperitoneal),the large polygonal tumor cells with transparent cytoplasm are arranged in a nest like manner, and the stroma is rich in small blood vessels. IHC findings **(B)**:Pax8 immunohistochemical staining of tumor cells is positive, indicating its renal origin.

**FIGURE 4:** Abdominal enhanced computed tomography (CT) findings at 6-month follow-up. Axial images from non-enhanced CT **(A)** to CT enhanced in arterial phase **(B)** and venous phase **(C)**. Non-enhanced CT **(A)** reveals the presence of a soft tissue density nodule in the surgical area (left para-abdominal aorta), CT enhanced in arterial phase **(B)** moderately enhanced nodules in the operative area, and decreased enhancement in venous phase **(C)**. No obvious abnormalities in either kidney are shown.

## Discussion

In this case, RCCC revealed extremely high FDG metabolic activity, which may be related to its pathological grade. The metabolic activity of FDG in renal clear cell carcinoma is related to pathological grade (2). Takahashi et al. found that highgrade clear cell renal cell carcinoma (ccRCC) showed higher metabolism than low-grade ccRCC, and high-grade on pathological nuclear grading was the most significant predictive value of SUV (3). According to the histological subtypes and the grade, high-grade ccRCC showed higher SUV than normal kidney tissues; in contrast, low-grade ccRCC did not show differences in the SUV when compared with normal kidney tissues (3). To explore the potential parameters from pre-operative ^18^F-FDG PET/CT that might associate with the World Health Organization/the International Society of Urological Pathology (WHO/ISUP) grade in ccRCC, Zhao Y. et al. revealed metabolic parameters of primary tumor SUVmax was significantly different between any two of the four different WHO/ISUP grades, except those between the WHO/ISUP grade 3 and grade 4. The optimal cutoff values to predict high WHO/ISUP grade for SUVmax was 4.15 (4). WHO/ISUP system is a universal RCC grading system. The higher the nuclear grading, the worse the tumor differentiation, the higher the invasiveness, and the worse the prognosis of patients. Therefore, the possible reason for the high SUVmax value of this patient is related to the low differentiation of the tumor.

RETRACTED

Remarkably, In this case, no abnormalities were found in either kidney *via* imaging or surgical exploration, findings that are likely suggestive of retroperitoneal renal tumor metastasis. Cancer of unknown primary site (CUPS) refers to primary tumors that cannot be detected by clinical, imaging, endoscopic, or other standard examination methods. CUPS accounting for 2.3–5% of all malignant tumors, of which nearly 80% can be presumed to be primary tumors *via* immunohistochemistry, molecular typing, genotype analysis, or other methods. In the remaining 20% of tumors, the origin of primary tissue cannot be determined (5, 6).

The pathogenesis of CUPS tumors is still unclear, Currently, two hypotheses have been formulated to describe their development. The first hypothesis states that all tumors have primary foci; however, the primary foci in CUPS tumors are too small or difficult to be detectable *via* existing clinical methods. As disease progresses or the accuracy of detection methods improves, primary foci will be found. The other hypothesis suggests that CUPS are a special type of tumors that exist independently (without primary foci) but are biologically similar (7).

Based on the clinical characteristics of CUPS tumors, patients are often referred for symptoms and signs related to metastases. To improve the diagnosis and evaluation of the tumors, it is important to obtain clues indicative of their primary tissue, therefore, it is necessary to comprehensively evaluate the patient’s history, tumor markers, imaging findings, and the tumor’s pathological type, immunohistochemistry, and gene expression profile and so on. Most tumors with unknown primary foci are adenocarcinomas (60%) and undifferentiated carcinomas (30%), while squamous cell carcinomas and/or transitional cell carcinomas (5–8%), neuroendocrine tumors (2–4%) and sarcomas (about 1%) are relatively rare (7, 8). The most commonly observed metastatic tumors with unknown primary foci are head and neck tumors, breast cancer, prostate cancer, pancreatic and biliary system primary tumors. The most common sites of metastasis include the lymph nodes, bone, liver, and lung (8). No prior case of RCCC with an unknown primary site has been reported in the literature.

RETRACTED

Large prospective clinical trials will be needed if we want to obtain conclusive evidence needed to improve treatment options for patients with tumors of unknown primary origin. According to current diagnosis and treatment guidelines, if a primary tumor can be reasonably presumed, the patient should be treated according to the specifications formulated for the presumed primary tumor, and the patient’s prognosis comparable to that of those with the specific type of primary tumor (7, 9). If no presumption can be made, patient prognosis varies and treatment includes empiric chemotherapy, palliative chemotherapy, and other supportive care. With the development of targeted therapy, successful cases of targeted therapy selected according to the molecular classification of tumors with unknown primary foci have been reported; however, no large-scale cohort study assessing the effectiveness of targeted therapy has reached a definitive conclusion (10–14). Immune checkpoint inhibitors have also been used to treat tumors of unknown primary origin, but only a subset of patients who have tumors with specific biological markers benefit from immunotherapy (15).

The diagnosis of occult tumors and those with an unknown clinical primary site comes with difficulties and challenges. Therefore, it is crucial to carefully read the film, take each patient’s history, obtain comprehensive laboratory results, and perform imaging and pathological examinations when evaluating such patients. PET/CT facilitates the whole-body assessment of patients. Some primary tumors may remain undetectable by PET/CT, but to transfer mode, scope, metabolic activity for overall evaluation, guiding the follow-up treatment measures, which have important significance, is also the primary focal unknown tumors guidelines recommended by the important assessment tool.

## Data availability statement

The original contributions presented in this study are included in the article/supplementary material, further inquiries can be directed to the corresponding author.

## Ethics statement

Written informed consent was obtained from the individual(s) for the publication of any potentially identifiable images or data included in this article.

## Author contributions

D-BZ conceived the project and wrote the manuscript. D-BZ, CC, and X-SL performed image post-processing and editing. D-BZ, YG, and Y-LW participated in the discussion and language editing. Z-JP reviewed the manuscript. All authors contributed to the article and approved the submitted version.
